The article "Perthamide C Inhibits eNOS and iNOS Expression and Has Immunomodulating Activity In Vivo" was retracted in 2019. Reasons: manipulated images; duplicated images; concerns about the data.

# Perthamide C Inhibits eNOS and iNOS Expression and Has Immunomodulating Activity In Vivo

**DOI:** 10.1371/journal.pone.0057801

**Published:** 2013-03-12

**Authors:** Mariarosaria Bucci, Anna Cantalupo, Valentina Vellecco, Elisabetta Panza, Maria Chiara Monti, Angela Zampella, Angela Ianaro, Giuseppe Cirino

**Affiliations:** 1 Department of Experimental Pharmacology, University of Naples Federico II, Naples, Italy; 2 Department of Biomedical and Pharmaceutical Sciences, University of Salerno, Fisciano (SA), Italy; 3 Department of Natural Products Chemistry University of Naples Federico II, Naples, Italy; University of Illinois at Chicago, United States of America

## Abstract

Here we have characterized perthamide C, a cyclopeptide from a Solomon Lithistid sponge *Theonella swinhoei*, which displays an anti-inflammatory/immunomodulatory activity. The study has been performed using the carragenan-induced mouse paw edema that displays an early (0–6 h) and a late phase (24–96 h). Perthamide C significantly inhibits neutrophils infiltration in tissue both in the early and late phases. This effect was coupled to a reduced expression of the endothelial nitric oxide synthase (eNOS) in the early phase while cyclooxygenase-1 and 2 (COX-1, COX-2), and inducible NOS (iNOS) expression were unaffected. In the late phase perthamide C reduced expression of both NOS isoforms without affecting COXs expression. This peculiar selectivity toward the two enzymes deputed to produce NO lead us to investigate on a possible action of perthamide C on lymphocytes infiltration and activation. We found that perthamide C inhibited the proliferation of peripheral lymphocytes, and that this effect was secondary to its metabolic activation *in vivo*. Indeed, in vitro perthamide C did not inhibit proliferation as opposite to its metabolite perthamide H.

In conclusion, perthamide C selectively interferes with NO generation triggered by either eNOS or iNOS without affecting either COX-1 or COX-2. This in turn leads to modulation of the inflammatory response through a reduction of vascular permeability, neutrophil infiltration as well as lymphocyte proliferation.

## Introduction

Within marine invertebrates, sponges have developed a highly complex immune system associated to the capacity to produce efficiently secondary metabolites as a defence mechanism. Moreover, sponges have provided a number of compounds exhibiting anti-inflammatory activity [1]. The cellular targets of these drugs are often different from those of non-steroidal anti-inflammatory drugs (mainly cyclooxygenase-1 or -2 inhibition) and in some cases relate to the inhibition of inflammatory gene transcription.

In our studies on bioactive compounds from sponges collected at Solomon Islands, [2] we found a single specimen of the sponge *Theonella swinhoei*, (Order Lithistida, Class Demospongia), as an extraordinary source of new metabolites. Analysis of the polar extracts afforded anti-inflammatory peptides such as the large library of perthamide C derivatives [3]–[6] and solomonamides A–B, [7] and anti-inflammatory sulfated sterols, solomonsterols A and B [8], potent agonists of the human nuclear receptor and xenobiotic sensor, pregnane-X-receptor (PXR) and new leads in the treatment of immune-driven inflammatory bowel diseases [9].

From a structural point of view, perthamide C has a peculiar unprecedented primary structure that comprises a 25-membered macrocycle with 6 out of the 8 residues constituted by unusual amino acids: γ-methylproline, *N* ^δ^-carbamoyl-β-OSO_3_Asparagine, *o*-tyrosine, d-ABU, *O*-methylthreonine, and the β-amino acid AHMHA (3-amino-2-hydroxy-6-methylheptanoic acid). Acute inflammatory response is characterized by an increase in vascular permeability and cellular infiltration leading to oedema formation as a result of extravasation of fluid and proteins, and accumulation of leukocytes at the inflammatory site. Following these changes, many other mechanisms are activated, contributing to the amplification of the inflammatory response and tissue damage, leading to the development of a more complex ‘scenario’ e.g. the chronic inflammatory reaction. Recently we have shown that perthamide C, among the different derivatives screened, significantly inhibited the inflammatory reaction in vivo [3]. Since perthamide C given systemically resulted active at very low dose e.g 0.3 mg/kg ip we have investigated in details the mechanism of this powerful anti-inflammatory activity.

## Materials and Methods

### Induction of edema in mouse paw

Male Swiss (CD-1; Harlan, Italy) weighing >30 g were divided into groups (n = 6 each group) and lightly anaesthetized with isoflurane. Each group of animals received subplantar injection of 50 µl of λ-carrageenan 1% (w/v) or 50 µl of saline in the left hind paw. Paw volume was measured by using an hydropletismometer specially modified for small volumes (Ugo Basile, Comerio, Italy) immediately before the subplantar injection and 2, 4, 6, 24, 48, 72 and 96 h thereafter. The same operator always performed the double-blind assessment of paw volume. The increase in paw volume was calculated as the difference between the paw volume measured at each time point and the basal paw edema. Each group of animals received 100 µl of perthamide C (0.3 mg/kg), or vehicle (polyethilenglycole, PEG) given i.p immediately before the injection of λ-carrageenan and 24 h thereafter. In a separate set of experiments dexamethasone (4 mg/kg) or vehicle (saline) were administered i.p.1 h prior λ-carrageenan injection and 24 h thereafter.

All procedures were performed according to Italian ministerial authorization (DL 116/92) and European regulations on the protection of animals used for experimental and other scientific purposes. The study was carried out in strict accordance with the recommendations in the Guide for the Care and Use of Laboratory Animals of the Italian Ministry of Health. The protocol was approved by the Committee on the Ethics of Animal Experiments of the University of Naples Federico II (Protocol Number: 2009/0047185). The paw edema was performed under enflurane anesthesia, and all efforts were made to minimize suffering.

### Myeloperoxidase (MPO) measurement in injected paws

Mice from different groups were euthanized with CO_2_ at different time points from λ-carrageenan or vehicle injection. Paws were cut, weighed and homogenized in 1 ml of hexadecyltrimethylammonium bromide (HTAB) buffer on ice by using a Polytron homogenizer (two cycles of 10 sec at maximum speed). After centrifugation at 10,000 rpm for 2 min, supernatant fractions were assayed for MPO activity as an estimate of cellular migration according to the method described in Posadas et al., 2004. Briefly, samples (20 µl) were mixed with phosphate buffer (180 µl) containing 1 mM O-dianisidine dihydrochloride and 0.001% hydrogen peroxide in a microtiter plate. Absorbance was measured at 450 nm, performing three readings at 30-s intervals. Calculation of MPO units was evaluated considering that 1 U MPO = 1 µmol H_2_O_2_ split and 1 µmol H_2_O_2_ gives a change in absorbance of 1.13×10^−2^ (change in absorbance = nm min).

### Western blot analysis

Paws were harvested from different groups of mice at different time points after λ-carrageenan or vehicle injection, and homogenized in modified RIPA buffer (Tris HCl 50 mM, pH 7.4, triton 1%, Na-deoxycholate 0.25%, NaCl 150 mM, EDTA 1 mM, phenylmethanesulphonylfluoride 1 mM, aprotinin 10 µg/ml, leupeptin 20 mM, NaF 50 mM) using a polytron homogenizer (two cycles of 10 sec at maximum speed) on ice. After centrifugation at 12,000 rpm for 15 min, protein concentration was determined by Bradford assay using BSA as standard (Bio-Rad Laboratories, Milan, Italy). 40 µg of the denatured proteins were separated on 10% SDS/PAGE and transferred to a PVDF membrane. Membranes were blocked in PBS-tween 20 (0.1%, v/v) containing 3% non fat dry milk for 1 hour at room temperature, and then incubated with anti-COX1 (1∶1000), anti COX-2 (1∶1000), anti-eNOS (1∶1000) or anti-iNOS (1∶500) overnight at 4°C. The filters were washed with PBS-tween 20 (0.1%, v/v) extensively for 30 min, before incubation, for 2 hours at 4°C, with the secondary antibody (1∶5000) conjugated with horseradish peroxidase antimouse IgG. The membranes were then washed and immunoreactive bands were visualized using an Enhanced Chemiluminescence Substrate (ECL; Amersham Pharmacia Biotech, San Diego, CA, USA).

### Preparation of cell suspension

Cell suspension was obtained as previously described [10]. Briefly, peripheral lymph nodes (PLN) (axillary, brachial, inguinal, cervical and mesenteric) were harvested from different groups of animals and at different time points from λ-carrageenan injection. Cells were pooled and prepared as single cell suspensions, by passing through a Nitex sieve (Cadisch Precision Meshes, London,UK) using a syringe plunger, and washed in sterile RPMI-1640 (Invitrogen Life Technologies, Paisley, UK). Monocytes were obtained by separation with Histopaque 10771 (Sigma, Milan, Italy). The cell suspensions obtained were used for the evaluation of the proliferative response to Concanavalin A (Con A).

### Proliferation assay

The MTT colorimetric assay, based on the ability of viable cells to reduce the yellow MTT (3-[4,5- dimethylthiazol-2-yl]-2,5-diphenyl tetrazolium bromide) salt to the blue MTT formazan product, was used to assess lymphocytes proliferation *in vitro*. Preliminary experiments determined that lymphocytes number and absorbance (570 nm) formed a linear relationship thereby providing a reliable assay for measurement of cell proliferation. PLN lymphocytes obtained from mice of each study group, were dispensed into 96-well plates at a density of 2×10^6^ cells per well in RPMI media containing streptomycin/penicillin (1%), sodium pyruvate (0.1%), 2-mercaptoethanol (0.1%) and foetal calf serum (10%) in a final volume of 150 µl and kept in an incubator at 37°C and in an atmosphere of, 5% CO_2_+95% air., To induce T cells proliferative responses cells were pulsed with Con A (5 µg/ml) for 72 h. In the last 4 h of incubation, 25 µl MTT reagent was added to each well. This step was followed by the addition of detergent reagent (100 ml per well) for 2 h to enable complete solubilisation of formazan product (plates kept in the dark). The absorbance of the samples was then measured using a microplate reader at 570 nm. Each treatment/assay was based on n = 6 replicate samples.

In a separate set of experiment we tested the biological activity of perthamide C on lymphocytes obtained from mice of the näive group. In this set of experiments, cells were pulsed for 72 h with Con A (5 µg/ml) in presence or absence of different concentrations (3-10-30 µM) of perthamide C.

### Sample preparation for mass spectrometry-based detection of perthamide C and H in mouse plasma

Plasma samples were collected from mice of each group at different time points after perthamide C administration. The clean-up procedure of plasma was performed by solid-phase extraction as previously described [11]. The Waters Sep-Pak Vac tC18 cartridges (50 mg) were initially washed with 2 ml ACN and then pre-conditioned with 5 ml of H_2_O containing 0.05%TFA and 2% HCOOH. 100 µl of ice plasma were put at 37 °C for 15 min and then diluted at 2 ml with H_2_O. Each sample was then applied onto the cartridge, the cartridge was washed with 2 ml of H_2_O containing 0.05% TFA and 2% HCOOH and the analytes were eluted using 100% ACN containing 0.05% TFA and 2% HCOOH. The eluted substances perthamides C and H were dried and the residues were dissolved in 100 µl of 100% ACN containing 0.05% TFA and 2% HCOOH. This procedure has been repeated 3 times for each of mice plasma at 0, 1, 4, 16 and 24 h, after each perthamide C administration.

Finally, in order to measure the recovery rate of extraction, the same procedure has also been carried out on blank samples spiked with both perthamides C and H and at different concentrations for 3 times; the recovery rate of the procedure is around 90%.

### RP-HPLC-MS/MS method for detection of perthamide C (1) and H (2) in mouse plasma

25 µl of the extracts were injected into the HPLC–MS system LTQ XL ThermoScientific equipped with Accelera 600 Pump and Accelera AutoSampler system. The mixture was separated on a Jupiter 5 µ C18 column from Phenomenex (150×2.00 mm) using a mobile phase consisted on H_2_O-0.05% TFA-2% HCOOH (eluent A) and ACN-0.05% TFA-2% HCOOH (eluent B). The eluents were linearly changed from 10% B to 70% B within 14 min; the columns flow rate was set at 200 µl/min. The mass-spectrometer was set to operate with an ESI ionization source in positive and negative mode. The capillary temperature was kept at 320 °C, the sheath gas flow rate and the auxiliary flow rate were set at 10 and 5, respectively. Instrument optimization was performed by direct infusion and manual tuning. Detection of perthamides C and H was performed using the selected reaction-monitoring mode (SRM). The transition of the deprotonated perthamide C molecule to its corresponding product ions was recorded at m/z 1066.5→1023.5 (-CONH) and m/z 1068.5→1025.5 (-CONH) and the transition of the protonated perthamide H molecule to its corresponding product ions was recorded at m/z 988.5→971.5 (-NH_3_). The collision energy used was set at 35.

As standard for calculating the relative percentage of these metabolites, several runs of samples containing perthamide C alone, perthamide H alone or the same concentration of perthamides C and H upon clean up procedure were also performed.

### Sponge material and isolation of perthamides C and H

*Theonella swinhoei* (order Lithistida, family Theonellidae) was collected on the barrier reef of Vangunu Island, Solomon Islands, in July 2004. Authorization to collection and exportation of sponge samples was released by Fisheries Department of Solomon Islands Government to IRD (Institut de Recherche pour le Dèveloppement, Polynesian Research Center on Island Biodiversity, BP529, 98713 Papeete, Tahiti, French Polynesia) in the frame of a research project entitled: ‘Coral Reef Initiative in The South Pacific’ (CRISP) ‘Biodiversité et substances marines actives’, volet Molécules actives, soutenu par l′Agence Française pour le Développement’, authorization IRD–AFDCZZ3012-02U. The sponge lyophilized material was kindly provided by Dr. Cecile Debitus, IRD. The sponge is not on the endangered and protected species list (CITES list, www.cites.org) and no specific permits were required for the described field studies. Taxonomic identification was performed by Dr John Hooper of Queensland Museum, Brisbane, Australia, where specimens are deposited under the accession number G3122662. Identity of perthamide C and H was established by comparison of their RM and mass data with those previously reported [6].

### Evaluation of ulcerogenic effect of perthamide C

Mice were randomly divided in three groups (n = 3 for each group) and deprived of food, but allowed to drink water at libitum, for 16 hours. Administration of perthamide C (0.3 mg/kg i.p.) indomethacin (20 mg/kg per os, 100 µl), or vehicle (PEG) were then performed. Indomethacin was used as positive control. Three hours after the drugs administration, mice were euthanized by an overdose of anesthetic and stomachs were harvested and washed in saline. A longitudinal incision along the greater curvature was performed and the stomachs were inverted over the index finger. Lesions were blindly evaluated macroscopically with an arbitrary score as follows:

0 = healthy; 1 = hyperemic

2 = lesions without blood

3 lesions with blood

### Drugs and Reagents

Bradford reagent was obtained from Bio-Rad (Bio-Rad laboratories, Segrate, Milan, Italy). The antibodies against COX-2, eNOS and iNOS were purchased from BD Transduction laboratories (U.S.A.). The antibody against COX-1 was from Santa Cruz Biotechnology, Inc (Milan, Italy). All other reagents and compound used were obtained from Sigma-Aldrich (Milan, Italy).

### Statistical analysis

Results were expressed as mean±s.e.m. The level of statistical significance was determined by one way ANOVA followed by Dunnett's test for multiple comparisons or t-test analysis where appropriate, using GraphPad Prism software (GraphPad Software Inc., San Diego, CA). Differences were considered statistically significant when p was less than 0.05. Each sample was processed at least in triplicate.

## Results

### Perthamide C inhibits MPO activity in carragenan-induced mouse paw edema

We have previously shown, that systemic administration of perthamide C significantly reduced both the early (0–6 h) and the late phase (24–96 h) of λ-carrageenan-induced paw edema displaying a dose-dependent (0.1, 0.3 and 1 mg/kg, i.p.) anti-inflammatory activity that reached almost 60% of oedema inhibition at the dose of 0.3 mg/kg [6].

To clarify the mechanism/s of action of perthamide C we firstly evaluated the MPO activity, as an index of neutrophil infiltration in response to λ-carrageenan injection. As shown in Figure1 A and B, λ-carrageenan injection induced a significative increase in neutrophil infiltration into the mouse paw. Administration of perthamide C reduced MPO activity as compared to vehicle group and this effect resulted statistically significant at 6 and 24 h after λ-carrageenan injection, when MPO activity reaches its highest levels (Figure1 A and B) [12].

**Figure 1:** Perthamide C reduces MPO activity in both phases of oedema. Paws were harvested at different time points 2-4-6 h (A) and 24-48-72-96 h (B) from each group of animals and processed in order to measure MPO activity. Values are expressed as mean±s.e.m. (*n* = 4–6 paws for each time point). ^*^P<0.05 ^**^P<0.01, ^***^P<0.001 vs S (saline), ° P<0.05, °° P<0.01 vs vehicle.

### Perthamide C reduces the expression of NOS but not COX isoforms

Next we evaluated if perthamide C administration was able to modify the expression levels of the constitutive enzymes eNOS and COX-1 as well as of their respective inducible isoforms, iNOS and COX-2. Thus, we performed western blot analysis on paw homogenates obtained from each groups of animals. As shown in figure 2 (panels A, B, C), during the early phase of edema both eNOS and COX-1 were expressed in total extracts obtained from saline- and λ-carrageenan-injected paw homogenates (Figure 2A and B). As expected, their inducible isoforms, iNOS and COX-2, were not detectable in this timeframe (data not shown). Systemic administration of perthamide C significantly reduced eNOS expression after 2 h and 4 h from λ-carrageenan injection (Figure 2A and B), while COX-1 expression was not modified by perthamide C treatment all throughout the early phase of edema (Figure 2A and C).

**Figure 2:** Western blot analysis of eNOS and COX-1 in the early phase of the paw edema. Expression of eNOS and COX-1 (A) were evaluated in total tissue extracts from paw homogenates obtained from mice treated with perthamide C, vehicle or saline at 2, 4 and 6 h following λ-carragenan injection (n = 4 paws for each treatment and time point). In panel B and C are shown the relative densitometric analysis °P<0.05, °°P<0.01 vs vehicle. Image is representative of three separate experiments.

We observed a different ‘scenario’ in the late phase of oedema following administration of perthamide C. In fact, as shown in figure 3 (panels A, B), systemic administration of perthamide C significantly reduced the expression of both NOS isoforms while it did not inhibit either COX-1 or COX-2 (Figure 4A and B).

**Figure 3:** Western blot analysis of eNOS and iNOS in the late phase of the paw edema. Expression of eNOS (A) and iNOS (B) were evaluated in paws homogenates obtained from mice treated with perthamide C, vehicle or saline at 24, 48, 72, 96 h following λ-carragenan injection. (n = 4 paws for each treatment and time point)^**^P<0.01vs saline, ° P<0.05, °° P<0.01, °°° P<0.001 vs vehicle. Image is representative of three separate experiments.

**Figure 4:** Western blot analysis of COX-1 and COX-2 in the late phase of the paw edema. Expression of COX-1 (A) and COX-2 (B) were evaluated in paws homogenates obtained from mice treated with perthamide C, vehicle or saline at 24, 48, 72, 96 h following λ-carrageenan injection. (n = 4 paws for each treatment and time point) ^*^P<0.05 ^**^P<0.01 vs saline. Image is representative of three separate experiments.

### Perthamide C inhibits Con-A induced cellular proliferation

Injection of λ-carrageenan in the hind paw causes activation and proliferation of T cells in the draining lymph nodes. Proliferation assays showed that lymphocytes harvested from control mice (mice receiving only λ-carrageenan) responded to Con A stimulation as compared to cells obtained from vehicle group (Figure 5). Treatment of mice *in vivo* with perthamide C (0.3 mg/Kg/i.p.) significantly suppressed the proliferative response to Con A of lymphocytes at all time points considered (4-48-96 hrs) as compared to the control group (Figure 5). Dexamethasone (4 mg/kg) was used as reference drug (Figure 5).

**Figure 5:** Proliferation assays on lymphocytes. Lymphocytes were obtained from PLN of control (vehicle) or perthamide C treated mice 4 h, 8 h or 96 h after λ-carrageenan edema induction. Values are means±SEM of three separate experiments with n = 5–6 mice. ^***^P<0.001 vs Naive+Con A; °°°P<0.001 vs CTL+Con A.

In a separate set of experiment we tested the biological activity of perthamide C *in vitro* on lymphocytes obtained from näive mice. Cells were pulsed for 72 h with Con A (5 µg/ml) in presence or absence of different concentrations (3-10-30 µM) of perthamide C (data not shown). Surprisingly, in contrast with the *ex-vivo* experiments, perthamide C added to the cells *in vitro*, did not modify Con A-induced cellular proliferation at any of the concentrations tested. Thus we hypothesized that the molecule we were using *in vitro* was probably subjected, *in vivo*, to a metabolic activation, most likely at the sulfate group on the *N* ^δ^-carbamoyl-β-OSO_3_Asparagine unit, thus acting as a pro-drug. To prove this hypothesis, we decided to test the effect of the desulfated perthamide C derivative, perthamide H, recently isolated by our research group from a deep re-investigation of the polar extracts of *Theonella swinhoei* [6]. As we hypothesized, the elimination of the sulfate group in perthamide C led to the active form of the molecule that was able to inhibit also *in vitro* and in a concentration-dependent manner, the Con A-induced proliferation of lymphocytes from näive mice (Figure 6).

**Figure 6:** Proliferation assays on lymphocytes harvested from näive mice. Perthamide H significantly inhibited, in a dose-dependent manner, Con A-induced proliferation of lymphocytes. Values are means±SEM of three separate experiments with n = 5–6 mice. ^***^P<0.001 vs basal (Bas);°°°P<0.001 vs Con A.

### Perthamide C is converted in vivo in its desulfated derivative, perthamide H

In order to measure the relative levels of perthamide C and H in mice plasma upon different time from each perthamide C administration, we resorted to a selective quantification of these metabolites by RP-HPLC-MSMS analysis. Plasma samples of three different mice collected at 1, 4 and 16 and 24 h from each perthamide C administration have been pre-cleaned by solid-phase extraction and the fractions eluted at 100% ACN have been submitted to RP-HPLC-MSMS runs operating in selected reaction monitoring (SRM) mode. Perthamide C shows two chromatographic peaks respectively at 12.25 min (MH^−^ at 1066.5) and at 22.50 min (MH^+^ at 1068.5); this behaviour was probably due to the charge state of *N* ^δ^-carbamoyl-β-OSO_3_Asparagine residue (Figure 7A and B). Perthamide H retention time is 12.33 min and its MH^+^ is 988.50 as expected (Figure 7A and B). The area of these three peaks has been integrated in each run and the results has been reported as relative percentage of the two metabolites (Figure 7C). At a starting point, 100% of perthamide C has been arbitrary set.

**Figure 7:** Chemical structure and LCMS runs of perthamide C and H. Panel A shows the chemical structure of perthamide C and H. Panel B shows one of the LCMS runs for detecting perthamides C and H in mice plasma samples using the selected reaction-monitoring mode (SRM). The peak at rt of 12.25 min corresponds to deprotonated perthamide C, the peak at rt of 12.33 min corresponds to protonated perthamide H, the peak at rt of 22.62 min corresponds to protonated perthamide C. Panel C shows the % of pertamides C and H detected by LCMS in mice plasma samples after 0, 1, 4, 16 and 24 h from each perthamide C administration.

It's noteworthy that, upon 1 h from each perthamide C administration, around 35% of this pro-drug has been desulfated giving rise to its active derivative perthamide H whereas, after 4, 16 and 24 h from each administration, decreasing levels of perthamide C and perthamide H have been detected.

### Perthamide C does not exert ulcerogenic action

In order to verify if perthamide C treatment could induce gastric lesions, a standard animal model for ulcerogenic activity was performed. As shown in Figure 8, perthamide C, at the dose that exerts anti-inflammatory action, did not induce any damage to gastric mucosa. Indeed, the score obtained from perthamide C treatment group (Figure 8B) was comparable to one obtained from vehicle group (Figure 8A). Conversely, administration of NSAID drug indomethacin, used as positive control, induced a massive ulcerogenic action (Figure 8C), as highlighted by the high score reached.

**Figure 8:** Perthamide C does not possess ulcerogenic action. Blindly arbitrary score was assessed as follows: 0 = healthy; 1 = hyperemic; 2 = lesions without blood; 3 lesions with blood; n = 3 for each group indomethacin was used as a control ulcerogenic drug. Pictures are representative of three different animals for each group of treatment.

## Discussion

In the present study we have investigated, in details, the molecular mechanism of the anti-inflammatory activity exhibited by perthamide C [3]. We have used to address this issue the λ-carrageenan mouse paw edema since due to its, sub-chronic nature it has allowed us to dissect the early event triggered within few hours from those that are deployed later within 3–4 days. In fact, the λ-carrageenan induced mouse paw edema as opposite to rats, produces a biphasic edema. In the first phase, which developed up to 6 h, edema is of low intensity, while in the second phase, after 24 h, edema is more pronounced and peaks at 72 h after λ-carrageenan injection [10], [12], [13]. Another important feature of this model is that, as the inflammation progresses, an increasing number of T cells infiltrate the draining lymph nodes of the λ-carrageenan-injected paws [10] thereby this model is also reminiscent of a typical type III immune reaction. In this reaction regional lymph nodes are the source of effector T cells that are postulated to extravasate at the site of antigen challenge and in turn, recruit and activate a variety of nonspecific inflammatory cells [14]. Perthamide C significantly inhibited the myeloperoxidase activity, a marker of neutrophil infiltration in tissue, in the early phase of the inflammatory reaction. This effect was coupled to a reduced expression of the endothelial nitric oxide synthase (eNOS) while COX-1, iNOS and COX-2 expression were unaffected. Thus, perthamide C inhibitory effect *in vivo* is fast on onset and its action is possibly linked to modulation of eNOS-derived NO. This feature well fit with the finding that, in this model, the increase in vascular permeability in the early phase is dependent upon eNOS-derived NO [15]. Most likely the modulation of perthamide C operated on eNOS is linked to its ability to bind hsp90 [16]. Indeed, hsp90 is instrumental for eNOS activation as elegantly demonstrated in the paper by García-Cardeña et al. [17].

Perthamide C reduced up to 96 h the expression of both NOS isoforms i.e. eNOS and iNOS without affecting COXs expression i.e. COX-1 and COX-2. This peculiar selectivity toward the two enzymes deputed to produce NO lead us to investigate on a possible action of perthamide C on lymphocytes infiltration and activation that is typical of the second phase of this animal model. Indeed, it is widely accepted that NO plays an important role in immunomodulation and neutrophil trafficking [18], [19]. In order to be consistent, we approached this issue by studying the proliferation of PLN lymphocytes harvested from mice receiving *in vivo* perthamide C. Lymphocytes challenged *in vitro* with Con A displayed a reduced proliferation demonstrating that the effect of perthamide C *in vivo* involves also these cellular population. This result suggested a potential immuno-suppressor activity for perthamide C.

In order to further investigate this effect a study was carried out in vitro on lymphocytes recovered from naïve mice. Surprisingly, in contrast with the *ex-vivo* experiments, perthamide C added *in vitro* to lymphocytes harvested from naïve mice, did not modify Con A-induced cellular proliferation at any of the concentrations tested. Therefore, we hypothesized that perthamide C was most likely subjected, *in vivo*, to a metabolic activation, probably at the sulfate group on the *N* ^δ^-carbamoyl-β-OSO_3_Asparagine unit, thus acting as a pro-drug. Our assumption was confirmed by the selective quantification of both metabolites by RP-HPLC-MSMS analysis carried out on plasma samples collected at different time points following each perthamide C administration *in vivo* to mice. This hypothesis was confirmed by the finding that desulfated perthamide C, namely perthamide H, did inhibit, in a concentration-dependent manner, the Con A-induced proliferation of lymphocytes harvested from naïve mice as opposite to perthamide C. The finding that perthamide C induces a state of immune-suppression acting *in vivo* only after metabolic activation represents an important outcome of our data since it give us a first insight into a structure/activity relationship.

The marine environment has proven to be a very rich source of extremely potent compounds that have demonstrated significant activities in anti-tumor, anti-inflammatory, analgesia, immuno-modulation, allergy and anti-viral assays. There are now significant numbers of very interesting molecules that have come from marine sources, or have been synthesized as a result of knowledge gained from a prototypical compound, that are either in or approaching Phase III clinical trials in cancer, analgesia and allergy. In conclusion we have defined an immunomodulatory activity of perthamide C in vivo and clarified that the action is due to its metabolite Perthamide H. Therefore this cyclic peptide could represent a new leading structure to develop therapeutics.

## References

[1] AlcarazMJ, PayáM (2006) Marine sponge metabolites for the control of inflammatory diseases. Current Opinion in Investigational Drugs7: 974–979.17117584

[2] Coral Reef Initiative in The South Pacific CRISP.

[3] FestaC, De MarinoS, SepeV, MontiMC, LucianoP, et al (2009) Perthamides C and D, two new potent anti-infiammatory cyclopeptides from a Solomon Lithistid sponge *Theonella swinhoei* . Tetrahedron 65: 10424–10429.

[4] SepeV, D'AuriaMV, BifulcoG, Ummarino R ZampellaA (2010) Concise synthesis of AHMHA unit in perthamide C. Structural and stereochemical revision of perthamide C. Tetrahedron 66: 7520–7526.

[5] FestaC, De MarinoS, SepeV, D'AuriaMV, BifulcoG, et al (2011) Perthamides C-F, potent human antipsoriatic cyclopeptides. Tetrahedron 67: 7780–7786.

[6] FestaC, De MarinoS, D'AuriaMV, MontiMC, BucciM, et al (2012) Anti-inflammatory cyclopeptides from the marine sponge *Theonella swinhoei* . Tetrahedron 68: 2851–2857.

[7] FestaC, De MarinoS, SepeV, D'AuriaMV, BifulcoG, et al (2011) Solomonamides A and B, New Anti-inflammatory Peptides from *Theonella swinhoei* . Organic Letters 13: 1532–1535.2134171510.1021/ol200221n

[8] FestaC, De MarinoS, D'AuriaMV, BifulcoG, RengaB, et al (2011) Solomonsterols A and B from *Theonella swinhoei*. The first example of C-24 and C-23 sulfated sterols from a marine source endowed with a PXR agonistic activity. J Med Chem 54: 401–405.2114196710.1021/jm100968b

[9] SepeV, UmmarinoR, D'AuriaMV, MencarelliA, D'AmoreC, et al (2011) Total synthesis and pharmacological characterization of solomonsterol A, a potent marine pregnane-X-receptor agonist endowed with anti-inflammatory activity. J Med Chem 54: 4590–4599.2159902010.1021/jm200241s

[10] IanaroA, O'DonnellCA, Di RosaM, LiewFY (1994) A nitric oxide synthase inhibitor reduces inflammation, down-regulates inflammatory cytokines and enhances interleukin-10 production in carrageenin-induced edema in mice. Immunology 82: 370–375.7959870PMC1414869

[11] BurkardI, von EckardsteinA, RentschKM (2005) Differentiated quantification of human bile acids in serum by high-performance liquid chromatography-tandem mass spectrometry. J Chromatogr B Analyt Technol Biomed Life Sci 826: 147–159.10.1016/j.jchromb.2005.08.01616182619

[12] PosadasI, BucciM, RoviezzoF, RossiA, ParenteL, et al (2004) Carrageenan-induced mouse paw oedema is biphasic, age-weight dependent and displays differential nitric oxide cyclooxygenase-2 expression. Br J Pharmacol 142: 331–338.1515554010.1038/sj.bjp.0705650PMC1574940

[13] IanaroA, XuD, O'DonnellCA, Di RosaM, LiewFY (1995) Expression of TGF-beta in attenuated Salmonella typhimurium: Oral administration leads to the reduction of inflammation, IL-2 and IFN-gamma, but enhancement of IL-10, in carrageenin-induced oedema in mice. Immunology 84: 8–15.7890306PMC1415173

[14] BlackCA (1999) Delayed type hypersensitivity: Current theories with an historic perspective. Dermatol Online J 5: 7.10673450

[15] BucciM, RoviezzoF, PosadasI, YuJ, ParenteL, et al (2005) Endothelial nitric oxide synthase activation is critical for vascular leakage during acute inflammation in vivo. Proc Natl Acad Sci U S A 102: 904–908.1564034810.1073/pnas.0408906102PMC545512

[16] MargarucciL, MontiMC, MencarelliA, CassianoC, FiorucciS, et al (2012) Heat shock proteins as key biological targets of the marine natural cyclopeptide perthamide C. Mol Biosyst 8: 1412–1417.2232711610.1039/c2mb05507d

[17] García-CardeñaG, FanR, ShahV, SorrentinoR, CirinoG, et al (1998) Dynamic activation of endothelial nitric oxide synthase by Hsp90. Nature 392: 821–824.958055210.1038/33934

[18] NiedbalaW, CaiB, LiewFY (2006) Role of nitric oxide in the regulation of T cell functions. Ann Rheum Dis 65: 37–40.10.1136/ard.2006.058446PMC179838617038470

[19] IanaroA, IalentiA, SautebinL, Di RosaM (1998) Nitric oxide inhibits neutrophil infiltration in the reverse passive arthus reaction in rat skin. Naunyn Schmiedebergs Arch Pharmacol 358: 489–495.982607210.1007/pl00005282

